The article "MiR-211-5p Inhibits the Biological Behaviors of Colorectal Cancer via SPARC-Related Growth Factor Pathways" was retracted in 2022. Reasons: concerns about the data; concerns about the images.

# MiR-211-5p Inhibits the Biological Behaviors of Colorectal Cancer via SPARC-Related Growth Factor Pathways

**DOI:** 10.7150/jca.60269

**Published:** 2022-03-21

**Authors:** Xiaoyu Wu, Yu Chen, Ya Zhu, Facai Cui

**Affiliations:** 1 Department of Clinical Laboratory, Henan Provincial People's Hospital, People's Hospital of Zhengzhou University, Zhengzhou, Henan, 450003, P. R. China.; 2 Department of Pathology, Affiliated Tumor Hospital of Zhengzhou University, Zhengzhou, Henan, 450008, P. R. China.

**Keywords:** colorectal cancer, growth factors, invasion, miR-211-5p, SPARC

## Abstract

Colorectal cancer (CRC) is a highly malignant cancer with poor prognosis. MiR-211-5p has been widely studied as an antioncogene; however, its function and mechanism in CRC are still unknown. This study aimed to investigate the expression patterns and biological implications of miR-211-5p in CRC. This study used quantitative real-time polymerase chain reaction to evaluate miR-211-5p expression in CRC cells and tissues. MiR-211-5p mimics were constructed to overexpress miR-211-5p in Lovo and SW480 cells. Tumor bioactivities of CRC, including cell proliferation, migration, invasion, and colony formation, were evaluated. The dual-luciferase assay was used to confirm the targeted relationship between miR-211-5p expression and secreted protein acidic and rich in cysteine (SPARC). In addition, Western blot analysis and immunohistochemical staining were used to measure SPARC, platelet-derived growth factor (PDGF), transforming growth factor β (TGF-β), and vascular endothelial growth factor (VEGF) expression levels. This study showed downregulated miR-211-5p expression in CRC cells and tissues, and this downregulation correlated with CRC progression. Meanwhile, miR-211-5p restrained CRC cell proliferation, colony formation, migration, and invasion. Mechanistically, SPARC-related growth factor pathways, including VEGF, PDGF, and TGF-β pathways, were upregulated in CRC tissues. Furthermore, SPARC acted as the target gene for miR-211-5p. Finally, SPARC overexpression suppressed the inhibitory effect of miR-211-5p on CRC cell progression. MiR-211-5p suppressed the invasion, migration, proliferation, and progression of CRC cells through sponging SPARC-related growth factor pathways.

## Introduction

Colorectal cancer (CRC), which mainly occurs in the junction of the rectum and sigmoid colon, is a highly malignant cancer with high incidence and mortality, killing almost 700,000 people annually 1-3. According to the World Health Organization reports, the incidence and mortality of CRC continue to increase 4. More than 60% of patients with CRC are in the final stage of the disease at the time of diagnosis due to the lack of typical clinical symptoms in the early stage of the disease 5, 6. Meanwhile, the abnormal growth and the excessive invasion of CRC cells mean that CRC can metastasize to other parts of the body via the blood and lymph systems, resulting in poor curative effects, high recurrence rates, poor prognosis, and high death rates 7. Therefore, it is important to elucidate the potential molecular mechanisms of CRC so as to determine effective targeted diagnostic strategies and therapies for CRC.

MicroRNAs (miRNAs) represent noncoding single-stranded RNAs that are 20-22 nucleotides in length 8, 9. They exert regulatory functions via directly combining with the 3′-UTRs of downstream target genes, thereby enhancing the degradation or translation inhibition of target genes 10, 11. Many studies have shown that miRNAs act as oncogenes or tumor suppressors in the pathogenesis of CRC, such as miR-541-3p 12, miR-324-3p 13, and miR142-5p 14. In recent years, miR-211-5p, a promising target gene, has been associated with the proliferation, metastasis, and development of melanoma 15, bladder cancer 16, and renal cancer 17. Chen found that miR-211-5p inhibited the proliferation, invasion, migration, and metastasis of triple-negative breast cancer through the direct targeting of SETBP1 18. In addition, Wang proved that miR-211-5p inhibited the metastatic behavior of renal cancer through the targeting of snail family transcriptional repressor 1^17^. However, the effects of miR-211-5p on the biological regulation of CRC are still unclear.

The secreted protein, acidic and rich in cysteine (SPARC), is part of the multifunctional secreted glycoprotein family; it participates in modulating cell-matrix interactions and cell functions 19, 20. SPARC exerts crucial effects during CRC growth, invasion, and metastasis by remodeling the extracellular matrix and facilitating epithelial-mesenchymal transition 21-23. More importantly, Liu found that patients with low SPARC expression had remarkably better disease-free survival and overall survival than patients with high SPARC expression 24. In addition, SPARC binds to several growth factors in a direct manner, including platelet-derived growth factor (PDGF), transforming growth factor β (TGF-β), and vascular endothelial growth factor (VEGF), which are related to the regulation of cancer hallmarks, such as angiogenesis, invasion, metastasis, and survival 25-28. These growth factors have also been reported to participate in cetuximab resistance, metastasis, CRC progression, and epithelial-mesenchymal transition 29-31. In addition, some studies reported SPARC as a major miR-211-5p target in inhibiting the biological properties of malignant cancers 32, 33. However, whether SPARC-related growth factor pathways have underlying roles in the effects of miR-211-5p requires further exploration.

Thus, this study aimed to discuss the expression patterns and biological implications of miR-211-5p in CRC. The potential roles of SPARC-related growth factor pathways (SPARC-VEGF, SPARC-PDGF, and SPARC-TGF-β) in the effects of miR-211-5p and CRC regulation were also illustrated. The results showed that miR-211-5p, as an antioncogene, had low expression in CRC tissues. A high miR-211-5p level was associated with favorable CRC prognosis *in vivo*, and miR-211-5p restrained proliferation, invasion, migration, and colony formation *in vitro*. Mechanically, miR-211-5p exerted its effects by sponging SPARC-related growth factor pathways.

## Materials and Methods

### Patients and samples

A total of 256 primary CRC tumor samples and matched non-carcinoma samples were obtained from patients who underwent surgical resection in Henan Provincial People's Hospital & People's Hospital of Zhengzhou University (Zhengzhou, China) between January 2016 and December 2018. 156 primary CRC tumor samples and matched non-carcinoma samples were preserved at -80 °C before RNA and protein extraction. At the same time, 100 pairs of tissues were fixed with 4% for immunohistochemistry. Data on patients' characteristics, including age, sex, tumor size, differentiation, lymph node metastasis, liver metastasis, and tumor-node-metastasis (TNM) classification, were collected. The study was approved by the ethics committee of the Henan Provincial People's Hospital & People's Hospital of Zhengzhou University.

### Cell culture and transfection

Human CRC-derived cells (HCT116, HCT8, Lovo, SW620, Caco2, and SW1463) were obtained from the Type Culture Collection of the Chinese Academy of Sciences (Shanghai, China). HIEC non-carcinoma human intestinal epithelial cells were obtained from the American Type Culture Collection (VA, USA) as internal and the A375 cells, the human melanoma cell line with low miR-211-5p expression, has been used in this study as external controls. The cells were stored in Gibco Dulbecco's modified Eagle Medium (Thermo Fisher Scientific, MA, USA) containing 10% fetal bovine serum (Life Technologies, Inc., NY, USA). All cell lines were cultured and grown at 37 °C and in the presence of 5% CO_2_. MiR-211-5p mimics or negative control (miR-NC) mimics were constructed by Guangzhou Rui Bo Biotechnology Co., Ltd. (Guangzhou, China) to evaluate miR-211-5p overexpression. The cells were considered processed using the NC mimics or miR-211-5p mimics when the cell confluence rate reached 50%-60% via Lipofectamine 2000 (Life Technologies, CA, USA). The interference efficiencies of the miR-211-5p mimics were investigated using qRT-PCR after 48 h. In addition, the SPARC agonist HY-P7291 (15 μmol/L) was used to upregulate SPARC levels.

### Cell proliferation assay

The CCK-8 assay (Dojindo Laboratories, Japan) was used to measure cell proliferation. After 48 h of transfection with NC mimics or miR-211-5p mimics, the cells were inoculated at a density of 2000 cells per well in 96-well plates, with 5 replicates. After 4 h of incubation in a humidity-controlled incubator, 10 μL of CCK-8 solution was added to each well. The proliferative activity was evaluated after 0, 12, 24, 48, and 72 h at a wavelength of 450 nm.

### Sphere-forming assay

Lovo and SW480 cells (500 cells/well) were inoculated into 6-well plates and incubated for 2 weeks following 24 h of transfection and incubation to investigate sphere-forming capacity. The medium was replaced every 2 or 3 days. The cells were rinsed twice using phosphate-buffered saline at designated times. The cell colonies were subsequently treated with 30 min of 0.5% crystal violet staining, and then images of tumor spheres were acquired.

### Wound-healing assays

The wound‐healing assay was used to measure cell migration capacity. SW480 and Lovo cells were inoculated into 24-well plates. Then, 48 h after transfection, scratch wounds were created at the cell layer using 10-μL tips when the cells reached 90% confluence. All cells were incubated in a serum-free medium for 48 h. The cells transferred to the wounded areas were photographed using an inverted-phase microscope.

### Transwell assay

The cell invasion capacity was measured using Transwell assay. First, 24 h after transfection, SW480 and Lovo cells were inoculated into the upper chamber at a density of 5 × 10^5^ cells/mL in 100 μL of serum-free medium, followed by culture for 24 h at 37°C. Then, the Transwell chamber was removed to eliminate the supernatant. Next, the cells that migrated or invaded the other side of the chamber were subjected to 4% paraformaldehyde fixation for 30 min as well as 0.1% crystal violet staining. The penetrated cells were photographed for analysis with Image Pro-Plus software.

### Dual-luciferase reporter assay

The miR-211-5p target was discerned using the TargetScan online software (http://www.targetscan.org). The mutant type (MUT) or wild type (WT) of the SPARC 3'‐UTR and putative binding sites of miR-211-5p in SW480 and Lovo cells were cloned into pGL3 vectors to assess whether SPARC was the effective target of miR-211-5p. The MUT and WT reporter 3'-UTRs of Wnt (Wnt-MUT and Wnt-WT, respectively) and SPARC (SPARC-MUT and SPARC-WT, respectively) were synthesized. The pGL3-SPARC 3'UTR-MUT or pGL3-SPARC 3'UTR-WT was co-transfected with miR-NC mimics or miR-211-5p mimics into cells using Lipofectamine 2000. Then, 48 h after incubation, the luciferase activity was measured using the FLUOstar equipment (Omega Engineering, Deckenpfronn, Germany).

### Western blot analysis

Following gross protein extraction in the tissues and CRC cells, the same amount of total protein (30 μg) was loaded into 10% acrylamide gel for sodium dodecyl sulfate sulfate-polyacrylamide gel electrophoresis, segmented by electrophoresis for 120 min, and then migrated to a polyvinylidene difluoride membrane for 100 min. The membrane was blocked and incubated with primary antibodies (anti-SPARC, anti-VEGF, anti-PDGF, anti-TGFβ, or anti-β-actin; all from Abcam, MA, USA) overnight at 4 °C. After being rinsed three times, the membrane was incubated with the secondary antibody at ambient temperature for 60 min. The protein expression was detected by electrochemiluminescence in the dark. Further, β-actin was used as the experimental internal control.

### Quantitative real-time polymerase chain reaction

Quantitative real-time polymerase chain reaction (qRT-PCR) was conducted following previous procedures 34. The major primer sequences were miR-211-5p (forward): 5′-GCGCTTGTCATCCTTCGCCT-3′; miR-211-5p (reverse): 5'-TGGTGTCGTGGAGTCG-3'; U6 (forward): 5′‐GCTTCGGCAGCACATATACTAAAAT‐3′; and U6 (reverse): 5′‐CGCTTCACGAATTTGCGTGTCAT‐3′. MiR-211-5p levels were measured using the PrimeScript miRNA RT-PCR Kit (TaKaRa Bio Inc., Isa Cit, Japan). The relative miR-211-5p expression was measured using the 2^-ΔΔCt^ technique.

### Immunohistochemical staining assay

To determine the protein expression levels of SPARC, VEGF, PDGF, and TGF-β, 15 CRC samples and matched normal samples were gathered from the patients. Subsequently, 4% routine dehydration and paraffin embedding were performed. The tissues were sliced into 4-mm-thick sections and incubated with the primary antibodies (anti-SPARC, anti-VEGF, anti-PDGF, anti-TGF-β, or anti-β-actin; all from Abcam, MA, USA) overnight at 4 °C. After being rinsed with PBS three times, the tissues were incubated with the secondary antibody at ambient temperature for 30 min. The nuclei were stained with diaminobenzidine coloring solution at ambient temperature for 15 min. The staining intensity and range were measured using the staining scores stipulated by Hu 35.

### Statistical analysis

Statistical analysis was performed using SPSS 23.0 (SPSS, Inc., IL, USA). Data were presented as mean ± standard deviation (SD). Differences were evaluated using Student *t* tests. Multiple group comparisons were analyzed using analysis of variance. The patient survival rates were measured using Kaplan-Meier survival analysis. A *P* value <0.05 indicated a statistically significant difference.

## Results

### Low miR-211-5p levels were related to poor prognosis in patients with CRC

A total of 156 primary CRC samples and matched noncarcinoma samples were gathered to measure miR-211-5p expression levels in CRC tissues. According to the qRT-PCR results, miR-211-5p levels significantly decreased in the CRC samples compared with the noncarcinoma samples (*P* < 0.05, Figure 1A). The clinical statistics of patients with CRC were gathered to further reveal the potential connection between miR-211-5p and CRC pathology. The results showed that patients with higher miR-211-5p levels had higher survival rates compared with those with lower miR-211-5p levels (*P* < 0.05, Figure 1B and 1C). The correlations between the miR-211-5p levels and the clinicopathological features of CRC were also investigated (Table 1). Increased miR-211-5p levels were remarkably related to poor prognosis, including tumor size (*P* < 0.001), TNM classification (*P* < 0.001), differentiation (*P* < 0.001), and liver metastasis (*P* < 0.05) (Table 1).

### SPARC, VEGF, PDGF, and TGF-β were underexpressed in CRC tissues

SPARC, VEGF, PDGF, and TGF-β are involved in the regulation of several CRC hallmarks. Therefore, the expression levels of SPARC, VEGF, PDGF, and TGF-β were detected by Western blot analysis and immunohistochemical staining assay. This study found that the protein levels of SPARC (*P* < 0.05, Figure 2A), VEGF (*P* < 0.05, Figure 2C), PDGF (*P* < 0.05, Figure 2E), and TGF-β (*P* < 0.05, Figure 2G) in CRC tissues were greater than those in adjacent normal tissues. Immunohistochemical staining intensity and range-based scoring revealed that the mean immunohistochemical scores of SPARC (*P* < 0.05, Figure 2B), VEGF (*P* < 0.05, Figure 2D), PDGF (*P* < 0.05, Figure 2F), and TGF-β (*P* < 0.05, Figure 2H) were significantly higher in the CRC tissue than in the adjacent normal tissues.

### MiR-211-5p suppressed the invasion, migration, proliferation, and colony formation of CRC cells

MiR-211-5p expression levels in CRC cells consistently increased than those in normal human colorectal mucosal cells (*P* < 0.05, Figure 3A). We transfected miR-211-5p mimics into Lovo and SW480 cells to investigate the biological functions of miR-211-5p during CRC progression. After miR-211-5p mimic transfection, the miR-211-5p levels in the Lovo and SW480 cells increased (*P* < 0.01, Figure 3B), suggesting that miR-211-5p mimic transfection was efficient. CCK-8 assay results showed markedly decreased CRC cell proliferation in the miR-211-5p mimic group compared with the NC mimic group (*P* < 0.05, Figure 3C and 3D). Compared with the NC mimic group, the miR-211-5p overexpression group showed significantly weakened colony formation ability in the CRC cells (*P* < 0.05, Figure 3E and *P* < 0.05, Figure 3F, respectively). Transwell assay results revealed that miR-211-5p downregulation obviously inhibited Lovo and SW480 cell invasion (Figure 3G and 3H). Similarly, the scratch assay results proved that Lovo and SW480 cell migration decreased in the miR-211-5p mimic-transfected cells (*P* < 0.05, Figure 3I and 3J).

### SPARC was the miR-211-5p target gene

TargetScan 7.2 was used to identify the miR-211-5p target gene. Interestingly, SPARC showed strong potential to be the miR-211-5p target (Figure 4A). The dual-luciferase reporter assay was performed to detect SPARC so as to further analyze the relationship between SPARC and miR-211-5p. Significant suppression was found when miR-211-5p mimics were transfected together with pGL3-SPARC-WT into the Lovo and SW480 cells (*P* < 0.05, Figure 4B and 4C), but pGL3-SPARC-MUT luciferase activity was not greatly influenced. SPARC expression levels within CRC cells were also analyzed by Western blot analysis to assess whether miR-211-5p regulated SPARC expression levels in CRC cells. The SPARC protein levels in the Lovo and SW480 cells were all downregulated by miR-211-5p mimics (*P* < 0.05, Figure 4D, 4E, and 4F). Meanwhile, SPARC-related growth factor pathways, including the VEGF, PDGF, and TGF-β pathways, were lower in the miR-211-5p mimic group than in the NC mimic group (*P* < 0.05, Figure 4D, 4E, and 4F).

### SPARC overexpression suppressed the influence of miR-211-5p downregulation in CRC cells

The SPARC agonist HY-P7291 was used to upregulate SPARC levels in Lovo and SW480 cells so as to explore whether the miR-211-5p-modulated regulation of the malignant biological properties of CRC cells was dependent on the targeting of SPARC. The expression levels of SPARC, VEGF, PDGF, and TGF-β increased after using the SPARC agonist in the Lovo cells (*P* < 0.05, Figure 5A and 5B) and SW480 cells (*P* < 0.05, Figure 5A and 5C). Further, the inhibiting effects of miR-211-5p in terms of malignant biological properties, including proliferation (*P* < 0.05, Figure 5D and 5E), colony-forming capacity (*P* < 0.05, Figure 5F and 5G), migration (*P* < 0.05, Figure 6A and 6B), and invasion (*P* < 0.05, Figure 6C and 6D), were reversed by the SPARC agonist.

## Discussion

CRC is a malignant cancer of the digestive tract; it is associated with a high incidence rate and poor quality of life. The abnormal growth and the excessive invasion of CRC cells are some of the leading reasons for CRC-related mortality 36. The present study showed that miR-211-5p expression was downregulated in CRC cells and tissues, and downregulated miR-211-5p levels predicted poor prognosis in patients with CRC. Meanwhile, miR-211-5p inhibited CRC cell invasion, migration, colony formation, and proliferation. Further, the expression of SPARC-related growth factor pathways, including the VEGF, PDGF, and TGFβ pathways, was found to be upregulated in CRC tissues. In addition, SPARC was identified as the miR-211-5p target gene, and SPARC overexpression restored the ability of miR-211-5p to suppress CRC cell progression. Therefore, it was concluded that miR-211-5p suppressed CRC progression by sponging SPARC-related growth factor pathways.

Mounting evidence suggests that miRNAs can serve as both oncogenes and anti-oncogenes, extensively participating in the occurrence and development of tumor cells 37-39. MiR-211-5p, which functions as a cancer suppressor gene, participates in tumor proliferation, invasion, and resistance 32, 40. The present study showed miR-211-5p downregulation in CRC samples, and this downregulation was associated with poor clinical outcomes and pathological characteristics, such as tumor size, TNM stage, differentiation, overall survival, and liver metastasis. Based on these findings, it was thought that miR-211-5p might have vital roles in the progression and prognosis of CRC. Regarding the function of miR-211-5p *in vitro*, miR-211-5p expression was found to be decreased in CRC cells compared with normal human intestinal epithelial cells. In addition, miR-211-5p overexpression after miR-211-5p mimic transfection was found to suppress Lovo and SW480 cell viability, invasion, migration, and colony formation, which was in accordance with the results of previous studies 41, 42.

SPARC has been reported to be involved in CRC invasiveness, extracellular matrix remodeling, epithelial-mesenchymal transition, angiogenesis, and tumor drug therapy response 43. Drev et al. found that the 5-year disease-free survival markedly decreased in patients with high SPARC levels compared with patients with low SPARC levels 23. Liu et al. found that low SPARC expression levels were associated with aggressive features in patients, such as bowel wall invasion, high carcinoembryonic antigen and Glucose polypeptide antigen 19-9 levels, and lymph node metastasis 24. In this study, SPARC expression levels in CRC tissues showed obvious differences from those in adjacent normal tissues *in vivo*. In addition, the luciferase reporter assay results showed that SPARC served as a direct target of miR-211-5p. Meanwhile, Western blot analysis results showed that SPARC protein levels were downregulated by the miR-211-5p overexpression. Further, the inhibitory effects of miR-211-5p in terms of malignant biological properties, including proliferation, colony-forming capacity, migration, and invasion, were reversed by the SPARC agonist. These results suggested that the miR-211-5p-mediated repression of SPARC might underlie the potential role of miR-211-5p in suppressing the malignant biological properties of CRC. In a related study, Liang suggested that the miR-211-5p/SPARC axis participated in the proliferation, migration, and invasion of papillary thyroid cancer 32, which was consistent with the results of the present study.

Multiple studies, including the present study, have shown that SPARC expression is related to malignant progression, but the mechanisms of the miR-211-5p/SPARC axis in tumorigenesis and metastasis are still unclear. This study suggested that SPARC could interact with growth factors, such as PDGF, VEGF, and TGF-β 44-46. Liang et al. showed that SPARC expression was obviously associated with VEGF expression in CRC, and SPARC-related VEGF was involved in the poor progression, invasion, and metastasis of CRC 47. Gorantla et al. reported that SPARC overexpression inhibited endothelial tube formation and induced programmed cell death by inhibiting the levels of pro-angiogenic molecules, such as VEGF, TGF-β, and PDGF, in endothelial cells 48. In this study, the expression levels of VEGF, PDGF, and TGF-β markedly decreased in CRC tissues compared with adjacent normal tissues. In addition, tumor biological activities were inhibited by miR-211-5p overexpression or inhibition of VEGF, PDGF, and TGFβ. Meanwhile, after using the SPARC agonist, miR-211-5p's inhibitory effects on the protein expression levels of VEGF, TGF-β, and PDGF were changed. Therefore, SPARC-related growth factor pathways, including SPARC-VEGF, SPARC-PDGF, and SPARC-TGF-β, might be involved in the underlying mechanisms of miR-211-5p-related inhibition of tumor biological activities.

In conclusion, it was found that miR-211-5p, which had decreased expression in CRC tissues, significantly influenced the adverse clinicopathologic features and prognosis of patients with CRC. Further, miR-211-5p was found to restrain CRC cell proliferation, invasion, migration, and colony formation by regulating SPARC-related growth factor pathways *in vitro*. This study was novel in revealing the function of the miR-211-5p/SPARC axis in CRC, hence providing a novel therapeutic target for human CRC.

## Figures and Tables

**Figure 1:** ** MiR-211-5p levels in CRC cells and tissues and their relationships with survival rates. (A)** MiR-211-5p levels were downregulated in CRC samples compared with matched noncarcinoma samples. **(B)** Thirty CRC cases were classified into low- and high-miR-211-5p-expression groups according to the average miR-211-5p expression level. **(C)** Cases with reduced miR-211-5p levels had enhanced cumulative survival rates. Values are expressed as mean ± SD. *P <0.05 indicated a statistically significant difference.

**Figure 2:** ** Expression levels of SPARC, VEGF, PDGF, and TGF-β in CRC tissues. (A)** SPARC expression measured through Western blot analysis. **(B)** SPARC expression measured through immunohistochemical staining assay. **(C)** VEGF expression measured through Western blot analysis. **(D)** VEGF expression measured through immunohistochemical staining assay. **(E)** PDGF expression measured through Western blot analysis. **(F)** PDGF expression measured through immunohistochemical staining assay. **(G)** TGF-β expression measured through Western blot analysis. **(H)** TGFβ expression measured through immunohistochemical staining assay. Magnification 200×. Data are expressed as mean ± SD. *P <0.05 indicated a statistically significant difference.

**Figure 3:** ** Increased miR-211-5p levels restrained the *in vitro* tumorigenesis of CRC cells. (A)** Reduced miR-211-5p expression levels in CRC cells compared with normal human epithelial cells. **(B)** MiR-211-5p was overexpressed after miR-211-5p mimic transfection. **(C and D)** Increasing miR-211-5p expression levels impeded cell proliferation, according to the CCK-8 assay. **(E and F)** Increasing miR-211-5p expression levels restrained clonal formation ability. **(G and H)** Increasing miR-211-5p expression levels suppressed migration capability, according to the Transwell assay. **(I and J)** Increasing miR-211-5p expression levels suppressed invasion capability, according to the scratch assay. The photomicrographs are typical images of SW480 and Lovo cells (400×). Values are expressed as mean ± SD. *P <0.05 indicated a statistically significant difference.

**Figure 4:** ** SPARC was the target pathway of miR-211-5p. (A)** TargetScan predicted an miR-211-5p binding site in the SPARC 3'-UTR. **(B and C)** Dual-luciferase reporter assay was conducted to detect SPARC luciferase activity. **(D, E, and F)** Expression levels of VEGF, SPARC, TGF-β, and PDGF in SW480 and Lovo cells were measured through Western blot analysis. Values are expressed as mean ± SD. *P < 0.01 compared with the si-NC group. #*P* < 0.01 compared with the si-LOXL1-AS1 group.

**Figure 5:** ** SPARC agonist suppressed the effects of miR-211-5p overexpression on cell viability and colony formation ability. (A, B, and C)** Expression levels of VEGF, SPARC, TGF-β, and PDGF in SW480 and Lovo cells were measured through Western blot analysis. **(D and E)** Viabilities of SW480 and Lovo cells were measured through CCK-8 assays. **(F and G)** Colony formation abilities of SW480 and Lovo cells were measured through colony formation assays. Typical images of SW480 and Lovo cells (400×). Values are presented as means ± SDs. *P <0.05 indicated a statistically significant difference.

**Figure 6:** ** SPARC agonist blocked the effects of miR-211-5p overexpression on cell migration and invasion. (A and B)** SW480 and Lovo cell invasion abilities were measured through Transwell invasion assays.** (C and D)** SW480 and Lovo cell migration abilities were measured through scratch assays. Typical images of SW480 and Lovo cells (400×). Data are denoted as means ± SDs. *P <0.05 indicated a statistically significant difference.

**Table 1:** Correlation between miR-211-5p level and clinicopathological characteristics

Characteristic	Patients (n)	miR-211-5p level		*χ* ^2^	*P*
		High	Low		
**Gender**				0.042	0.838
Male	102	74	28		
Female	54	40	14		
**Age, year**				0.878	0.349
<50	98	68	30		
≥50	58	36	22		
**Body mass index, kg/m^2^**				0.220	0.639
<23	79	35	44		
≥23	77	37	40		
**Tumor size, mm**				30.195	0.001
≤5	65	49	16		
>5	91	28	63		
**Differentiation**				7.523	0.006
Well/Moderate	72	45	27		
Poor	84	34	50		
**TNM stage**				9.479	0.002
0 & I & II	47	25	22		
III & IV	109	30	79		
**Lymph node metastasis**				4.501	0.034
Negative	67	42	25		
Positive	89	29	60		
**Liver metastasis**					
Negative	66	45	21	5.784	0.016
Positive	90	44	46		

TNM: tumor-node-metastasis.

## Abbreviations

CRC: Colorectal cancer
SPARC: secreted protein acidic and rich in cysteine
PDGF: platelet-derived growth factor
TGF-β: transforming growth factor β
VEGF: vascular endothelial growth factor
MUT: mutant type
WT: wild type
TNM: tumor-node-metastasis
qRT-PCR: Quantitative real-time polymerase chain reaction
